# Effects of kinematic complexity and number of muscles on musculoskeletal model robustness to muscle dysfunction

**DOI:** 10.1371/journal.pone.0219779

**Published:** 2019-07-24

**Authors:** M. Hongchul Sohn, Daniel M. Smith, Lena H. Ting

**Affiliations:** 1 The George W. Woodruff School of Mechanical Engineering, Georgia Institute of Technology, Atlanta, Georgia, United States of America; 2 Wallace H. Coulter Department of Biomedical Engineering, Emory University and Georgia Institute of Technology, Atlanta, Georgia, United States of America; 3 Department of Rehabilitation Medicine, Division of Physical Therapy, Emory University, Atlanta, Georgia, United States of America; The Ohio State University, UNITED STATES

## Abstract

The robustness of motor outputs to muscle dysfunction has been investigated using musculoskeletal modeling, but with conflicting results owing to differences in model complexity and motor tasks. Our objective was to systematically study how the number of kinematic degrees of freedom, and the number of independent muscle actuators alter the robustness of motor output to muscle dysfunction. We took a detailed musculoskeletal model of the human leg and systematically varied the model complexity to create six models with either 3 or 7 kinematic degrees of freedom and either 14, 26, or 43 muscle actuators. We tested the redundancy of each model by quantifying the reduction in sagittal plane feasible force set area when a single muscle was removed. The robustness of feasible force set area to the loss of any single muscle, i.e. general single muscle loss increased with the number of independent muscles and decreased with the number of kinematic degrees of freedom, with the robust area varying from 1% and 52% of the intact feasible force set area. The maximum sensitivity of the feasible force set to the loss of any single muscle varied from 75% to 26% of the intact feasible force set area as the number of muscles increased. Additionally, the ranges of feasible muscle activation for maximum force production were largely unconstrained in many cases, indicating ample musculoskeletal redundancy even for maximal forces. We propose that ratio of muscles to kinematic degrees of freedom can be used as a rule of thumb for estimating musculoskeletal redundancy in both simulated and real biomechanical systems.

## Introduction

Musculoskeletal models have been used to explore motor redundancy, demonstrating how muscle dysfunction impacts motor output. For example, the effects of muscle weakness have been explored to understand gait deficits in cerebral palsy [1] and stroke [2, 3], as well as to predict outcomes of interventions that alter muscle function such as strengthening, tendon transfer [4], or botulinin toxin injection [5]. However, the kinematic description of the skeletal system can greatly alter the predicted force output of muscle activation [6], while the number of modeled muscles can alter model sensitivity to variations in muscle properties [7]; generally, studies of muscle dysfunction have not considered the effect of model complexity.

Studies show conflicting results about the robustness in biomechanical capabilities of human limb musculoskeletal models to the loss of a single muscle. Removing a single muscle typically has little effect on the ability of a lower-limb musculoskeletal model to reproduce experimentally-measured joint torques during walking [8, 9]. Specifically, single muscle dysfunction can be compensated for by other muscles, as the upper and lower bounds on feasible muscle activation ranges span 0 to 1 across most of the gait cycle in most muscles. In contrast the feasible muscle activation ranges for a finger model of static force production were tightly bounded [10]. The same study also showed that static force production in both the human finger and leg can be dramatically compromised by single muscle loss, as indicated by the vulnerability in the feasible force set that characterizes the maximum endpoint force in all directions [11, 12].

Such discrepancies in modeling studies of musculoskeletal redundancy likely arise from differences in the number of kinematic degrees of freedom, number of muscles, and the task examined. Planar leg models with three kinematic degrees of freedom (DoFs) and either nine [13] or fourteen [10, 14] muscles have been used to investigate muscle function. Three-dimensional (3D) models range from a human finger model with four DoFs and seven muscles [11], to cat hindlimb models with seven DoFs and 31 muscles [15], and human lower leg models with 23 DoFs and 92 muscles [9]. Such models have been used to examine variety of motor tasks including standing balance, pedaling, isometric force generation, and walking. To our knowledge, there has been no study systematically examining how various levels of model complexity alter the robustness of the musculoskeletal system to muscle dysfunction within a single motor task.

To resolve differences in prior literature, here we sought to explicitly examine how the kinematic complexity and the number of independent muscle actuators in a musculoskeletal model alter the effects of muscle dysfunction on motor output for a single task. We compared the robustness of six human leg models to single muscle loss during static force production. The simplest planar model was similar to that used in Kutch and Valero-Cuevas (2011) [10], and the most complex 3D model was similar to that used in Simpson et al. (2015) [9]. Because our main objective was to directly compare the same measure of musculoskeletal redundancy across models of varying complexity, including the sagittal plane model, we restricted our analyses to endpoint force production in the sagittal plane. We show that robustness to muscle dysfunction decreases with the number of kinematic DoFs and increases with the number of muscle actuators, and can greatly affect conclusions about how muscle strength affects biomechanical function.

## Materials and methods

We compared the robustness of six musculoskeletal models of the human leg to single muscle loss during static force production in the sagittal plane. Models with low kinematic complexity (Lo-DoF) had three planar DoFs; models with high kinematic complexity (Hi-DoF) had seven non-planar degrees of freedom. For each kinematic model, we simulated 14 muscle groups (Lo-Mus), 26 (Int-Mus) muscle groups, and 43 independently controlled muscles (Hi-Mus). For each model, we computed robustness and sensitivity to muscle dysfunction as the area of the feasible force set preserved and reduced after the loss of any muscle (or muscle group), respectively. As a further measure of redundancy, we tested whether feasible muscle activation ranges at maximal force production were constrained or allowed a range of muscle activation levels. All models, data, and codes for reproducing our results are available from the Dryad Digital Repository: https://doi.org/10.5061/dryad.28pj314 [16].

### Musculoskeletal models

We used a generic 3D musculoskeletal model of human leg (OpenSim Gait2392 [17]) with seven kinematic DoFs (Hip: 3, Knee: 1, Ankle: 2, MTP: 1) and 43 muscles/muscle compartments (Table 1). Posture was set to that resembling the mid-phase of pedaling at which experimental and model-based feasible force sets has been identified previously [13]: 48° hip flexion, 0° hip adduction, 0° hip rotation, 53° knee flexion, 33° ankle plantarflexion, 0° subtalar inversion, 0° metatarsophalangeal (MTP) joint angle. We selected such posture as it pertains to maximal force generation during pedaling, and also avoids singularity in joint torque to endpoint force mapping. The pelvis was fixed in space and the endpoint defined as the location of the MTP joint, which was pinned to the ground via a gimbal joint.

**Table 1:** Muscles included in each model and their abbreviations.

Muscle Name	Abbreviation					
	“Lo-Muscle” Model		“Int-Muscle” Model		“Hi-Muscle” Model	
		14 muscles		26 muscles		43 muscles
*Gluteus medius anterior*	1		1	GMED1	1	GMED1
*Gluteus medius middle*	2		2	GMED2	2	GMED2
*Gluteus medius posterior*	3	GMedMin	3	GMED3	3	GMED3
*Gluteus minimus anterior*	4		4	GMIN1	4	GMIN1
*Gluteus minimus middle*	5		5	GMIN2	5	GMIN2
*Gluteus minimus posterior*	6		6	GMIN3	6	GMIN3
*Semimembranosus*	7		7	SEMIMEM	7	SEMIMEM
*Semitendinosus*	8	HAM	8	SEMITEN	8	SEMITEN
*Biceps femoris long head*	9		9	BFLH	9	BFLH
*Biceps femoris short head*	10	BFSH	10	BFSH	10	BFSH
*Sartorius*					11	SAR
*Adductor longus*	12	ADDL	12	ADDL	12	ADDL
*Adductor brevis*					13	ADDBREV
*Adductor magnus superior*					14	ADDMAG1
*Adductor magnus middle*					15	ADDMAG2
*Adductor magnus inferior*					16	ADDMAG3
*Tensor fascia latae*	17	TFL	17	TFL	17	TFL
*Pectinueus*					18	PECT
*Gracilis*					19	GRAC
*Gluteus maximus anterior*	20		20	GMAX1	20	GMAX1
*Gluteus maximus middle*	21	GMax	21	GMAX2	21	GMAX2
*Gluteus maximus posterior*	22		22	GMAX3	22	GMAX3
*Iliacus*	23	ILIAC	23	ILIAC	23	ILIAC
*Psoas*					24	PSOAS
*Quadratus femoris*					25	QUADF
*Gemellus*					26	GEM
*Piriformis*					27	PIRI
*Rectus femoris*	28	RF	28	RF	28	RF
*Vastus medialis*	29		29	VM	29	VM
*Vastus intermedius*	30	VAS	30	VI	30	VI
*Vastus lateralis*	31		31	VL	31	VL
*Gastrocnemius medial head*	32	GAS	32	MEDGAS	32	MEDGAS
*Gastrocnemius lateral head*	33		33	LATGAS	33	LATGAS
*Soleus*	34	SOL	34	SOL	34	SOL
*Tibialis posterior*	35	TP	35	TP	35	TP
*Flexor digitorum longus*					36	FLEXD
*Flexor hallucis longus*					37	FLEXH
*Tibialis anterior*	38	TA	38	TA	38	TA
*Peroneus brevis*	39	PBREV	39	PBREV	39	PBREV
*Peroneus longus*					40	PLONG
*Peroneus tertius*					41	PTERT
*Extensor digitorum longus*					42	EXTD
*Extensor hallucis longus*					43	EXTH

Each gray box for the “Lo-Muscle” Model indicates grouped muscles.

To systematically alter model complexity, we created six models from the generic OpenSim model that varied in numbers of kinematic DoF and muscles. Two levels of kinematic DoF complexity were used: all seven DoFs allowing 3D motion (Hi-DoF) and three sagittal plane flexion/extension DoFs at the hip, knee, and ankle (Lo-DoF). Three sets of muscles were used: the complete set of 43 muscles with independent control (Hi-Muscle), a reduced set of 26 muscles with independent control (Int-Muscle), and a reduced set of 26 muscles with 14 independent muscles/muscle groups (Lo-Muscle) (see Table 1), similar to Kutch & Valero-Cuevas (2011). For completeness, we also created an alternative intermediate set of muscle actuators (alt-Int-Muscle) that used all 43 muscle models but with only 26 31 independent controls. The results from alt-Int-Muscle did not affect the general message of the results and were therefore not reported (data available [16]).

### Feasible force sets

To compute feasible force sets representing the bounds in biomechanical capability of each model in generating static endpoint forces, we first defined a linear mapping between endpoint force and muscle activation:

$$R\;F_{act}^{M}\;\overset{⃑}{a}=J^{T}{\overset{⃑}{F}}_{end}={\overset{⃑}{\tau }}_{net},$$ (1)

where ***R*** is the moment arm matrix, $F_{act}^{M}$ is a diagonal matrix of the maximum active muscle force each muscle can produce for the given muscle posture, $\overset{⃑}{a}$ is the muscle activation vector, ***J*** is the Jacobian matrix that maps the end-point wrench into the resultant net joint torques (${\overset{⃑}{\tau }}_{net}$), and ${\overset{⃑}{F}}_{end}$ is the endpoint wrench vector, however designated as force as moments were constrained to be zero. The moment arm matrix ***R*** was obtained by OpenSim [17], communicated via an application programming interface (API) to MATLAB (Mathworks, Inc., Natick, MA, USA). The API was used to extract muscle tendon unit length, maximum isometric force, optimal fiber length, tendon slack length, and pennation angle at optimum fiber length for each muscle. These parameters and the force-length relationship from an existing Hill-type muscle model [18] were used to calculate the active muscle force matrix, $F_{act}^{M}$ [19]. To calculate the Jacobian, ***J***, we converted the OpenSim leg model to Neuromechanic software [20], which has a function for numerically calculating the Jacobian between specified points on the model.

We computed each feasible force set in the joint torque space, utilizing the linear relationship between endpoint force to net joint torque (Eq 1), because the Jacobian transpose for some models was not invertible to define a direct linear mapping between muscle activation and endpoint force. As in prior studies [21, 22], we used *linprog*.*m* in MATLAB to find $\overset{⃑}{a}$ that maximizes ${\overset{⃑}{\tau }}_{net}$ in each of the torque directions for 300 evenly spaced unit wrench vectors, ${\hat{F}}_{dir}$, in the sagittal plane:

$$\max_{\overset{⃑}{a}}\;\left|{\overset{⃑}{\tau }}_{net}\cdot {J^{T}\hat{F}}_{dir}\right|\;s.t.\;{\overset{⃑}{\tau }}_{net}||{J^{T}\hat{F}}_{dir}\;and\;\overset{⃑}{0}\leq \overset{⃑}{a}\leq \overset{⃑}{1}.$$ (2)

Note from Eq 1 that ${\overset{⃑}{\tau }}_{net}=R\;F_{act}^{M}$, and in above equation (Eq 2) that $J^{T}{\hat{F}}_{dir}$ is the projection of ${\hat{F}}_{dir}$ into torque space. Thus, the goal was to find a vector $\overset{⃑}{a}$ that maximizes the magnitude of ${\overset{⃑}{\tau }}_{net}$ along the direction of vector $J^{T}{\hat{F}}_{dir}$.

Maximal endpoint force, ${\overset{⃑}{F}}_{end}^{MAX}$, in each specified direction was computed by multiplying the relative magnitude of the actual torque vector to the unit force vector:

F⃑endMAX=‖τ⃑net‖‖JTF^dir‖F^dir. (3)

Each feasible force set was defined as the convex polygon that contained all sagittal plane components of ${\overset{⃑}{F}}_{end}^{MAX}$ as determined by the *convhull*.*m* function in MATLAB [22]. Although our feasible force set was comprised of only the sagittal plane forces, optimization (Eq 2) was solved with six-dimensional wrench vectors (${\hat{F}}_{dir}$) that had non-zero elements only for the sagittal plane force components. Also note that solution to above optimization for 3D models (Hi-DoF) must satisfy the net torque requirements (Eq 1) in all of the seven DoFs, including the three non-sagittal DoFs. Activations of muscles that were grouped in the Lo-Muscle Model (Table 1) were constrained to be the same.

### Robustness and sensitivity of feasible force set to single muscle loss

The impact of muscle dysfunction on motor output was determined by examining the effect of single muscle loss on feasible force set area in the sagittal plane [10]. Single muscle loss was simulated by constraining a single muscle’s activation level to zero and recalculating the feasible force set. Robustness and sensitivity of the feasible force set to single muscle loss was defined as the percent area that was preserved and lost by loss of a given muscle, respectively. By definition, *sensitivity*+*robustness* = 100%, such that an increase in muscle redundancy would be indicated by an increase in feasible force set *robustness* to single muscle loss and a decrease in feasible force set *sensitivity* to single muscle loss.

While we quantified and report both robustness and sensitivity to single muscle loss for each muscle in each model, we focused our analyses of robustness and sensitivity to two different types of single muscle loss: *general* and *specific* single muscle loss, respectively. To characterize general capability of the model to maintain motor output against any potential muscle loss of muscle function, we first focused on examining the robustness of each feasible force set to *general* single muscle loss, defined as the percent area of the feasible force set unaffected by the loss of any single muscle (Fig 1, green hashed areas), i.e. the intersection of all the feasible force sets resulting from specific single muscle loss. To compare feasible force set area and robustness across models, sagittal plane feasible force set areas were normalized to that of the simplest model Lo-Muscle/Lo-DoF.

**Fig 1:** Sagittal plane feasible force sets (FFSs) and their robustness and sensitivity to general single muscle loss. Feasible force sets (blue regions) represent the set of all biomechanically feasible force vectors that each model can produce at the endpoint, defined as the location of the MTP joint, assuming independent activation of individual muscles. The area of each feasible force set in the sagittal plane is normalized with respect to that from the Lo-Muscle/Lo-DoF model. Robustness and sensitivity of each feasible force set to general single muscle loss is quantified by the percentage of the feasible force set occupied and unoccupied, respectively, by the robust region (green hashed regions), defined as the set of forces unaffected by the loss of any single muscle. Feasible force sets in the top row (A, B, and C) were created with three planar DoFs (Lo-DoF), while feasible force sets on the bottom row (D, E, and F) are from models with seven, three-dimensional DoFs. Feasible force sets in the left column (A and D) are from models with a grouped, reduced set of muscles (Lo-Muscle), totaling 14. The feasible force sets in the middle column (B and E) are from models with an independent, reduced set of 26 muscles (Int-Muscle). The feasible force sets in the right column (C and F) are from models with a set of 43 independent muscles (Hi-Muscle). In each panel, nMusc and nDoF stands for number of muscles and number of degrees of freedom, respectively.

To characterize muscle-specific deficit at motor output, on the other hand, we focused on examining the sensitivity of each feasible force set to *specific* single muscle loss, i.e. sensitive region of the feasible force set that gets lost after dysfunction of a particular muscle (Fig 2, see inset, blue area). In addition, we examined how grouping muscles, a simplification often used in literature (e.g. Lo-Muscle model in our study), affects the feasible force set sensitivity to single muscle (group) loss.

**Fig 2:** Sensitivity and robustness of feasible force sets (FFSs) to specific single muscle loss. The inset (top right) shows the preserved (green) and lost (blue) area of the feasible force set when one muscle, VL, is removed in the Hi-Muscle/Lo-DoF model. The sensitivity of the feasible force set to specific single muscle loss is defined as the percent reduction of the feasible force set to loss of each individual muscle. Results are presented for all muscles in ascending orders for sensitivity (blue bars) and descending order for robustness (green bars) for each model (each panel). The distribution of feasible force set sensitivity to single muscle loss is quantified by a box plot (right side of each graph) and the values corresponding to each quartile are extended across each graph.

### Feasible muscle activation ranges at maximum force

To quantify redundancy in muscle space, we identified feasible ranges of activation in individual muscles for maximal force in each model in all sagittal plane force directions. We used linear programming to find the upper and lower bounds on each individual muscle’s activation [15] at each maximum endpoint forces ${\overset{⃑}{F}}_{end}^{MAX}$:

$$J^{T}{\overset{⃑}{F}}_{end}^{MAX}=R\;F_{act}^{M}\;\overset{⃑}{a},$$ (4)

The minimum and maximum values of each element of $\overset{⃑}{a},$ *a*_*i*_ were identified one at a time, allowing the remaining elements of $\overset{⃑}{a}$ to vary (from 0 to 1) as necessary,

$$\min_{\overset{⃑}{a}}a_{i}\;s.t.\;J^{T}{\overset{⃑}{F}}_{end}^{MAX}=R\;F_{act}^{M}\;\overset{⃑}{a}$$ (5)

$$\min_{\overset{⃑}{a}}-a_{i}\;s.t.\;J^{T}{\overset{⃑}{F}}_{end}^{MAX}=R\;F_{act}^{M}\;\overset{⃑}{a}.$$ (6)

Feasible muscle activation ranges were classified based on their width as *determined* (width = 0), *undetermined* (width > 0), or *unconstrained* (width = 1).

## Results

Intact feasible force sets were qualitatively similar to previous reports in humans [10, 13] and animals [21] in that they were roughly elliptical with the axis approximately aligned with the limb axis, and the largest forces directed distally from the endpoint (Fig 1, blue areas). In general, feasible force set area increased with the number of independent muscles (Fig 1, left to right), and decreased with number of kinematic degrees of freedom (Fig 1, top to bottom); the decrease in Hi- vs. Lo-DoF models was less pronounced in the Int-Muscle and Hi-Muscle models.

### Effect of model complexity on robustness to general single muscle loss

Feasible force set robustness to the loss of any single muscle increased with the number of independent muscles (Fig 1, green areas). Lo-Muscle model feasible force sets were the smallest and least robust to general single muscle loss (Fig 1A and 1D), while the Int-Muscle model feasible force sets were slightly larger and significantly more robust to general single muscle loss (Fig 1B and 1E). Hi-Muscle model feasible force sets had the largest area and were the most robust to general single muscle loss (Fig 1C and 1F). However, larger feasible force set areas did not always correspond to greater robustness to general single muscle loss (compare Fig 1A and 1E).

Lo-DoF models were more robust than Hi-DoF models to the loss of any single muscle, but these differences were much less pronounced as the number of independent muscles increased (Fig 1, percent decrease from Lo-DoF to Hi-DoF: Lo-Muscle: 90%, Int-Muscle: 36%, and Hi-Muscle: 6%). Feasible force set robustness to general single muscle loss was approximately 50% in Hi-Muscle models, regardless of the number of DoFs.

### Effect of model complexity on sensitivity to specific single muscle loss

Feasible force set sensitivity to loss of a single muscle (Fig 2, blue bars) decreased as the number of independent muscles increased (Fig 2, left to right) and was higher in Hi-DoF models (Fig 2, top to bottom). The effects of increasing DoFs was less pronounced in models with more independent muscles.

The maximum sensitivity of the feasible force set to the loss of a single muscle decreased sharply as the number of independent muscles increased. In Lo-Muscle/Lo-DoF and Lo-Muscle/Hi-DoF, the maximum single muscle loss sensitivities were 68% and 75%, respectively, both due to loss of VAS (abbreviation defined in Table 1, Fig 2A and 2D). However, the maximum sensitivity was about 3 times smaller in Hi-Muscle models (26% for both Lo- and Hi-DoF) due to loss of VL (Fig 2C and 2F).

The loss of particular muscles had drastically different effects on the feasible force set in Hi-DoF versus Lo-DoF models. For example, the Int-Muscle/Lo-DoF feasible force set was least sensitive to PBREV (0% sensitivity, Fig 2B) while Int-Muscle/Hi-DoF feasible force set was most sensitive to PBREV (50% sensitivity, Fig 2E).

### Grouping muscles increases sensitivity to single muscle loss

Feasible force set sensitivity to single muscle (group) loss increased dramatically when muscles were grouped. Sensitivity to loss of a muscle group in the Lo-Muscle model (e.g. Fig 3A (VAS) and 3D (HAM), blue areas) was much larger than the sensitivity to loss of the corresponding muscles in the Int-Muscle model (e.g. Fig 3B (VM, VI, and VL) and 3E (SEMIMEM, SEMITEN, and BFLH), blue areas). Only when all of the participating muscles were removed from the Int-Muscle model, was the remaining feasible force set equivalent to loss of the grouped muscle in the Lo-Muscle models (e.g. compare Fig 3A with 3C, and 3D with 3F). More than half of the muscles to which the Hi-Muscle model feasible force sets were most sensitive (top ≈20% in Fig 2C and 2F) were part of grouped muscles in the Lo-Muscle models (Fig 2A and 2D). The sum of the sensitivities to loss of the independent muscles within each group was approximately equal to the sensitivity of the loss of the entire group (e.g. compare Fig 3A with 3B, and Fig 3D with 3E). Discrepancies were due to slight differences in total feasible force set area causing differences in sensitivity to single muscle loss across models (e.g. SOL: 11.6% vs 12.2% sensitive in Lo/Lo vs Int/Lo Models, Fig 2A and 2B).

**Fig 3:** Feasible force set sensitivity and robustness to loss of Vasti and Hamstring muscles in grouped and ungrouped muscle models. Feasible force set sensitivity and robustness to single muscle loss of selected grouped muscles from Lo-Muscle, (A) VAS and (D) HAM. Feasible force set sensitivity and robustness to single muscle loss of the independent muscles from Int-Muscle corresponding to the grouped muscle from Lo-Muscle, (B) VM, VI, and VL and (E) SEMIMEM, SEMITEN, and BFLH. (C) and (F) Feasible force set sensitivity and robustness to the loss of the group of corresponding independent muscles from Int-Muscle (“grouped muscle loss”).

### Wide feasible muscle activation ranges for maximal force production

The degree of possible variation in a single muscle’s activity for maximal force production varied widely across muscles and force directions, ranging from being fully determined to fully unconstrained. Feasible muscle activation ranges at maximum force for each muscle (Fig 4) varied between 0 and 1, (Fig 4, inner and outer circles, respectively) during maximum force production across all sagittal plane directions. Feasible muscle activation ranges were *determined* to a single value in some directions (Fig 4A, width = 0, green solid lines), while *undetermined* in other directions (Fig 4A width>0, green shaded area), delineating the range of muscle activation for which it is possible to produce a maximal force in that direction.

**Fig 4:** Feasible muscle activation ranges for maximum forces for selected muscles. (A) Feasible muscle activation ranges for the maximum sagittal plane forces for an example muscle, MEDGAS, in the Hi-Muscle/Hi-DoF model. The inner black circle represents a muscle activation of zero and the outer black circle represents a muscle activation of one, i.e. maximal activation. Each radial line between the two black circles corresponds to the feasible muscle activation range for a maximum force along that direction in the sagittal plane (right: anterior, up: superior). The minimum and maximum feasible activations for the maximum force in each direction in the sagittal plane are indicated in green. Feasible muscle activation ranges are either *determined*, i.e. with only one feasible solution, indicated by a solid green line (e.g., see posterior force directions in A), *undetermined*, i.e. with more than one feasible solution, indicated by a green shared area between the lines representing minimum and maximum feasible muscle activations (e.g., see anterior forces in A), or *unconstrained* (a subset of *undetermined*), i.e. where all solutions are feasible, represented by green shared areas that span completely from the inner to the outer black circles (e.g., see inferior forces in A). (B) Feasible muscle activation ranges for selected muscles (columns) in six models of varying complexity (rows).

Only the hip-knee bi-articular muscles were fully *determined* in maximum sagittal plane force production (Lo-Muscle: 3 of 14 muscles, Int-Muscle: 5 of 26 muscles, Hi-Muscle: 7 of 43 muscles). These muscles were generally constrained to zero activation for about half of the directions (e.g. Fig 4, left column, anterior-superior directions) and to full activation for the remaining directions (e.g. Fig 4, left column, posterior-inferior directions). Differences in these muscles’ constrained activations across models were minor.

Most muscles were fully constrained in some maximum sagittal plane force directions, but unconstrained in others (e.g. Fig 4, VAS and TA). These muscles were often constrained to have zero activation in some directions, and maximal activation in the opposite direction. However, they could adopt a range of activation level in other directions (e.g. Fig 4, VAS and TA).

In some cases, undetermined feasible muscle activation ranges were *unconstrained* (width = 1, green shaded area covers the entire area between the inner and outer circles) meaning that activation of muscle can be any value between 0 and 1 during maximum force production in that direction. The percentage of sagittal plane force directions with undetermined feasible muscle activation ranges in at least one muscle was high in all models and only slightly increased due to increased model complexity (Lo-Muscle/Lo-DoF: 86%, Hi-Muscle/Hi-DoF: 89%). Most undetermined feasible muscle activation ranges were also unconstrained.

Grouping muscles greatly limited the width of the unconstrained feasible muscle activation ranges and affected the directions for which they were constrained or unconstrained (e.g. Fig 4, VAS). The range of directions in which muscles were unconstrained varied from most directions (e.g. TA) to approximately half of the directions (e.g. VAS).

## Discussion

Our work suggests that debates about the degree of musculoskeletal redundancy in the musculoskeletal systems likely arise from difference in model complexity in prior studies. We show that the impact of simulated muscle dysfunction using musculoskeletal models depends greatly on kinematic complexity and numbers of independent muscle groups. Removing non-planar DoFs increases model redundancy, decreasing the effect of muscle dysfunction on motor output. By contrast, reducing the number of independent muscles or muscle groups decreases musculoskeletal redundancy, amplifying the effects of muscle dysfunction. As a rule of thumb, a ratio using the number of muscles-to-joints may be useful to compare the redundancy of musculoskeletal models as well as real biomechanical systems.

Removing a kinematic DoF from a musculoskeletal model either increases the maximum endpoint force in a given direction, or leaves it unchanged, leading to an increase in redundancy. Conversely, if a DoF is created or unlocked, maximum endpoint force magnitudes can only decrease or remain the same. Accordingly, we found that feasible force sets from planar models were more robust to the loss of a single muscle than feasible force sets from 3D models with the same set of muscles. One of the most impactful simplifications was locking the two non-planar DoFs of hip rotation. In the planar model, only the contributions of hip muscle to sagittal plane forces remained, without regard for their out-of plane contributions to endpoint force.

Removing a muscle from a musculoskeletal model either decreases the maximum endpoint force in a given direction or leaves it unchanged, leading to a decrease in redundancy. When a muscle is removed, it decreases the torque capacity of one or more DoFs, decreasing the maximum endpoint force in all direction limited by the torque capacity at those DoFs, and thus muscle redundancy. Conversely, adding a muscle allows all maximum forces limited by the torque capacity the DoF the muscle crosses to increase in magnitude. Accordingly, we found that maximum force production in models with fewer independently-controlled muscles was less robust to than models with more muscles but the same DoFs; grouping muscles drastically reduced the robustness of the feasible force sets.

As a rule of thumb, the higher the ratio of muscle to kinematic DoFs, the greater the musculoskeletal redundancy, reducing the effects of muscle dysfunction. We further propose that muscles-to-DoFs ratio in the form of (# *of muscles*)/(# *of kinematic DoF*+1) can be a useful measure for estimating musculoskeletal redundancy; this form accounts for the fact that minimum number of tension-only actuators (e.g. muscles) to fully actuate a N-DoF serial manipulator (e.g. leg) is N+1 [23, 24]. For example, our modified OpenSim leg model [17]–the most complex model used in this study–had muscles-to-DoFs ratio of 5.4 and demonstrated ample redundancy. This model was similar to that used to demonstrate that almost any single muscle can be completely activated or deactivated while still generating joint torques in human walking [8, 9]. In contrast, the model with smallest number of muscles and higher kinematic complexity had a muscle-to-DoFs ratio of 1.8, and was very sensitive to muscle dysfunction, similar to prior results [10]. A human index finger model verified in cadaveric studies had a muscles-to-DoFs ratio of 1.4 [10–12], and demonstrated high sensitivity to muscle loss. While our analysis was based on leg models, muscles-to-DoFs ratio of most actuated subparts of the human musculoskeletal system, including arm [25], fingers [6, 12], and spine [26, 27]fall within the range we examined (Table 2). Therefore the number of muscles and DoFs may explain discrepant results regarding the degree of redundancy in musculoskeletal systems. However, the muscle-to-DoFs ratio is only a rule of thumb and care needs to be taken when examining its relationship to paricular aspect of the degree of redundancy, which will depend on the specific anatomy, posture, and the actions of muscles crossing the kinematic DoFs [28–31].

**Table 2:** Redundancy in representative models of subpart of the locomotor system.

Modeled subpart	Total	Mean±std # of muscles per DoF	Minimum # of muscles per DoF	Redundancy measure
Lower extremity [32]	7 DoF ^a)^ 43 muscles	17±8.7	4	5.4
Upper extremity [25, 33]	7 DoF ^b)^ 50 muscles	22±3.4	18	6.3
Thumb [6]	5 DoF 8 muscles	6.0±2.2 ^c)^	2	1.3
Index finger [12]	4 DoF 7 muscles	5.3±0.4	5	1.4
Neck (Cervical spine) [26]	6 DoF 26 muscles	7.7±0.9	6	3.7
Lumbar spine [27]	3 DoF ^d)^ 210 (22 ^e)^) muscles	204±2.8 (22)	202 (22)	52.5 (9.1)

a) Translational DoF of patella constrained as a function of knee flexion angle.

b) Simplified to only include DoF proximal to wrist, i.e., excluding hand and fingers. Scapula and clavicle DoF constrained as a function of shoulder DoF.

c) Considering also actions of muscles via proximal and terminal tendon slips.

d) DoF of 5 lumbar intervertebral joints constrained to be proportion of the total lumbar movement in each rotational DoF.

e) If 210 muscle fascicles modeled are grouped into 22 muscle groups (11 on each side), assuming common neural inputs to each group.

Although we limited our comparison of musculoskeletal model redundancy to a static, maximal force generation in the sagittal plane, our results likely extend to non-planar, dynamic, and submaximal motor tasks. Human leg feasible force set is expected to have highest aspect ratio in the sagittal plane [13], where the shape and orientation may be sensitive to model parameters. However, our previous work in a cat hindlimb model that had complexity (muscles-to-DoFs ratio: 3.9) within the range of human limb models examined here suggests that the overall shape and magnitude of feasible force set in models with such level of complexity are not sensitive to model architectural and morphological parameters [21]. We made dataset and linear models for generating three-dimensional feasible force set available for use [16] in examining feasible force set in other motor tasks where force production in non-sagittal plane can be important, e.g. for stabilitization in the frontal plane during standing balance [34] or locomotion [35]. Motor tasks requiring submaximal forces, on the other hand, are generally expected to confer greater robustness, and thus a higher degree of musculoskeletal redundancy. Owing to linear construction of our models (Eq 1), the feasible forces we calculated encapsulate force production at any level [36]. Impact of muscle dysfunction in force production task at 50% of maximum level, for example, can thus be readily depicted by comparing the robust area to the smaller feasible force set, i.e., geometrically scaled by 50% in all directons. Redundancy in muscle space, as quantified by feasible muscle activation ranges, are expected to be greater in all models, as constained bounds in most muscles tend to emerge near maximal force production [15, 37]. We have indeed found that feasible muscle activation ranges for all muscles in all models were wider at 50% of maximum force, with many feasible muscle activation ranges that were fully determined at maximum force in all directions becoming fully unconstrained at 50% of maximum force in all directions (data available in [16]), further supporting our findings of wide feasible muscle activation ranges for maximal force production. Incorporating dynamics in a submaximal task, wide feasible muscle activation ranges have been demonstrated in a complex model of human gait [9], indicating that single muscles could be removed without loss of function [8, 38]. Similarly, a three-dimensional upper extremity model demonstrated that during manual wheechair propulsion, substantial reduction in strength of individual muscles can be compensated by other muscles [39].

Finally, our results highlight that musculoskeletal biomechanics are often insufficient to determine muscle activity even in maximal force production tasks, allowing for variations in neural strategies for muscular force production. The sensitive region of a feasible force set to loss of a single muscle comprises all the force directions and magnitudes where the muscle is necessary to generate the maximal force [15]. However, feasible muscle activation ranges, which explicitly identify the degree of possible variation in a single muscle’s activity [40], were largely unconstrained in many cases, demonstrating the biomechanical latitude that the nervous system has when selecting muscle activation patterns for the same motor task. As such, multiple functional criteria such as stability, resistance to fatigue, or generalizability [41–43], rather than single optimality [38, 44–49], may underlie the diversity in muscle activation patterns observed across individuals with varying motor training or neurological health [50].
